RETRACTED

# Clinical practice of epidermal growth factor receptor-tyrosine kinase inhibitor targeted drugs combined with gadolinium oxide nanoparticles in the treatment of non-small cell lung cancer

**DOI:** 10.1080/21655979.2021.2009969

**Published:** 2021-12-25

**Authors:** Xuan Zhou, Ting Jin, Likun Wang, Erlin Zhao, Xuyang Xiao

**Affiliations:** a Department of Thoracic Surgery, The First Affiliated Hospital of Jinzhou Medical University, Jinzhou, China; b Department of Rehabilitation, The First Affiliated Hospital of Jinzhou Medical University, Jinzhou, China

**Keywords:** Epidermal growth factor receptor-tyrosine kinase inhibitor (EGFR-TKI), hyaluronic acid-gadolinium sesquioxide-nanoparticles (HA-Gd2o3-NPs), non-small cell lung cancer (NSCLC), clinic

## Abstract

It was to explore the clinical efficacy and safety of epidermal growth factor receptor-tyrosine kinase inhibitor (EGFR-TKI) targeted drugs combined with hyaluronic acid-gadolinium sesquioxide-nanoparticles (HA-Gd2O3-NPs) in non-small cell lung cancer (NSCLC). In this study, 70 patients with stage IV EGFR mutant NSCLC diagnosed in the First Affiliated Hospital of Jinzhou Medical University were selected. They were randomly divided into the combined group (35 cases) and the control group (35 cases). HA-Gd2O3-NPs were prepared by hydrothermal polymerization, and combined with EGFR-TKI in the clinical treatment of NSCLC. The results showed that HA-Gd2O3-NPs were spherical with a uniform particle size of about 124 nm. The NSCLC survival rate of the combined group was 37.2 ± 5.3% under 6 Gy X-ray irradiation, and that of the control group was 98.4 ± 12.6% under 6 Gy X-ray irradiation. The total effective rate of the control group (20%) was significantly lower than that of the study group (42.86%) (*P <* 0.05). The one-year survival rate of the combined group (94%) was significantly higher than that of the control group (75%) (*P <* 0.05). The median progression-free survival (PFS) in the control group was 8 months, and that in the combined group was 12 months, with statistical difference (*P <* 0.05). EGFR-TKI targeted drugs combined with HA-Gd2O3-NPs can significantly improve the clinical efficacy of stage IV EGFR mutant NSCLC patients and benefit their survival.

## 1. Introduction

The incidence rate and mortality rate of lung cancer ranks first in China’s malignant tumors. According to the global cancer epidemiology statistics in 2020, the number of new cases of lung cancer worldwide is 2 million 207 thousand, second only to breast cancer. The number of deaths reached 1.796 million, ranking first among all cancer species [1]. In 2020, there were 816,000 new cases of lung cancer and 715,000 deaths in China. Among them, 80–85% of patients are non-small cell lung cancer (NSCLC) [2]. Due to the high invasiveness of NSCLC and the lack of effective early screening program, 70% of lung cancer patients in China are in advanced stage when diagnosed, and the 5-year survival rate is about 15% [3–5]. Clinical radiotherapy is a recognized non-invasive method for the treatment of cancer, which can be the same as the early treatment of lung cancer and alleviate the pain of metastatic lesions.

RETRACTED

In recent years, with the development of molecular typing technology, people have a new understanding of the biological mechanism of the occurrence and development of NSCLC, found several special subtypes of driving genes such as epidermal growth factor receptor (EGFR), adenolymphoma kinase (ALK), threonine protein kinase, and developed corresponding targeted drugs, opening the era of accurate treatment of NSCLC [6]. At this year’s annual meeting of the American Society of Clinical Oncology (ASCO), targeted therapy of NSCLC is still a hot topic explored by scientists and clinical experts [7]. It is suggested that epidermal growth factor receptor-tyrosine kinase inhibitor (EGFR-TKI) should be used for local treatment in patients with EGFR mutation positive brain metastasis of NSCLC. EGFR-TKI is recognized as the standard treatment for EGFR mutation positive and initial metastatic treatment NSCLC. The targeted nature of such drugs has good clinical value in reducing patients’ toxic and side effects and improving their clinical treatment effect. At present, it has been confirmed by a large number of clinical research results [8,9]. For NSCLC patients with EGFR mutation, drug resistance is the main obstacle to the effective treatment of targeted drug EGFR-TKI.

Nano rare earth materials (such as nano rare earth oxides) have been highly concerned and widely used in fluorescent materials, magnetic materials, hydrogen storage materials, and catalytic carrier materials because of their special nano effects [10]. At present, the preparation methods of nanoscale rare earth oxides include hydrothermal method, precipitation method, and sol–gel method. Gadolinium (GD) nanoparticles can be used as sensitizing materials for ionizing radiation, enhance X-ray and particle beam irradiation, and can be used as radiotherapy sensitizer for NSCLC cells [11]. Gadolinium oxide nanoparticles have good biocompatibility in NSCLC cells. In this experiment, hyaluronic acid gadolinium trioxide nanoparticles (HA-Gd2O3-NPs) were synthesized by hyaluronic acid, passivation molecule, and gadolinium chloride. Compared with normal lung tissue cells with low expression of EGFR, these new nanoparticles can specifically target lung cancer cells with high expression of EGFR, and can also realize active targeting to tumor cells through surface modified ligands Accurate drug delivery [12]. HA-Gd2O3-NPs, as a drug carrier, specifically targets EGFR mutant NSCLC cells and efficiently releases loaded drugs, which provides a new method for EGFR mutant lung cancer patients to overcome the resistance of EGFR-TKI.

RETRACTED

At present, some studies suggest that targeted combined with nanotherapy can improve the clinical efficacy of NSCLC, but its safety and effectiveness are not clear, so the efficacy of different combined methods remains to be explored. The innovation of this paper is to prepare HA-Gd2O3-NPs and combine them with EGFR-TKI in the clinical treatment of NSCLC, in order to explore the clinical efficacy and safety of their combined effect and provide reference basis for clinical treatment.

## 2. Research object and research method

### 2.1 Research object

Seventy patients with stage IV EGFR mutant NSCLC diagnosed in the First Affiliated Hospital of Jinzhou Medical University from 15 May 2020 to 15 May 2021 were selected. They were randomly divided into combined group (35 cases) and control group (35 cases). There were 42 males and 28 females, aged 40–75 years. This experiment has been approved by the committee of the First Affiliated Hospital of Jinzhou Medical University. The patients and their families understood the research situation and signed the informed consent form.

Inclusion criteria:(1) over 18 years old; (2) Physical situation score (PS score) is less than or equal to 2 points; (3) NSCLC was confirmed by histopathological examination; (4) Lung cancer was determined as stage IV according to TNM staging 8 issued by Union for International Cancer Control (UICC); (5) The expected survival time is more than 3 months; (6) EGFR mutation (+); (7) there is at least one tumor focus that can be analyzed; (8) No contraindications of targeted therapy and good compliance; (9) There was no history of lung surgery.

Exclusion criteria: (1) organ dysfunction, diseases of the blood system, diseases of the immune system, combined malignant tumors of other parts, and severe infection; (2) Those with combined mental diseases; (3) Patients with drug allergy; (4) Recently, patients used drugs that interfered with the experimental treatment plan.

### 2.2 Preparation of HA-Gd2O3-NPs

HA-Gd2O3-NPs was prepared by hydrothermal polymerization [13]. 0.15 g hydrated gadolinium chloride (Sigma-Aldrich, USA) and 0.25 g sodium acetate (Suzhou Huahang Chemical Technology Co., Ltd., China) were dissolved in 25 mL ethylene glycol (Shandong Xima Supply Chain Management Co., Ltd., China), and stirred vigorously at 80°C overnight, and cooled to room temperature. 0.3 g transparent acid (Guangzhou Charlan Biotechnology Co., Ltd, China) and 0.5 g sodium hydroxide (Guangzhou Charlan Biotechnology Co., Ltd., China) were added, stirred vigorously for 60 min, and then the solution was transferred to the reaction still. The reaction temperature was set to 180°C, heated for 4 h, cooled to room temperature, filtered, dialyzed, and lyophilized to obtain HA-Gd2O3-NPs. Figure 1 shows the preparation flow chart of hyaluronic acid gadolinium trioxide nanoparticles.

RETRACTED

**Figure 1.** Preparation flow chart of hyaluronic acid gadolinium trioxide nanoparticles

### 2.3 Hyaluronic acid gadolinium trioxide nanoparticles test and analysis

The phase composition of hyaluronic acid gadolinium trioxide nanoparticles was tested by Rigaku D/max-2500PC X-ray diffraction (XRD) (Rigaku corporation, Japan). The test conditions were as follows: CuKa radiation source, working voltage 40 kV, working current 200 mA, and scanning rate 4 (°)/min. The morphology of hyaluronic acid-gadolinium trioxide-nanoparticles was observed by S-4700 field emission scanning electron microscope (Hitachi, Japan). Hitachi H-800 transmission electron microscope (TEM) (Hitachi, Japan) was used to observe the morphology and particle size distribution of hyaluronic acid-gadolinium trioxide-nanoparticles.

After the prepared nano suspension was centrifuged (12,000 r/min, 20 min, 4°C), the supernatant was collected and filtered by microporous membrane. The content of EGFR-TKI in the supernatant was determined as the free dose in the system, and then the entrapment efficiency of drug loaded nanoparticles was calculated according to the formula.

(1) $$Entrapment\;efficiency\left(\;\%\right)=\left(total\;dosage-free\;dosage\right)/total\;dosage\times 100\%$$

### 2.4 Treatment methods

Control group: patients with EGFR-TKI resistance, only chemotherapy, intravenous infusion of 500 mg/(m^2^·d) pemetrexed disodium (Sichuan Huiyu Pharmaceutical Co., Ltd., China). 25 mg/(m^2^·d) cisplatin (Kunming Guiyan Pharmaceutical Co., Ltd., China). Each chemotherapy cycle is 21 days, 4 to 6 treatment cycles (according to the patient recovery and tolerance).

Combined group: after EGFR-TKI resistance occurred, the patients were first treated with three-dimensional conformal radiation therapy. After plastic fixation, the patients were simulated and localized under CT machine. The primary pulmonary lesions and intrapulmonary metastases were irradiated with linear accelerator 6 MV-X ray: the total dose was 58–64 Gy, 2 Gy/time, 5 times/week. The total dose of whole-brain radiotherapy was 34 ~ 42 Gy, 2 Gy/time, 5 times/week. The total dose of bone metastases was 32 Gy, 3 Gy/time, 5 times/week. Dose control: mean lung dose ≤ 20 Gy, both lungs V20 ≤ 30%, both lungs V5 ≤ 65%, spinal cord ≤ 45 Gy. EGFR-TKI targeted drug therapy, oral gefitinib tablets 250 mg/day (AstraZeneca Pharmaceutical Co., Ltd., China), once a day.

RETRACTED

### 2.5 Cell activity test of non-small cell carcinoma

Logarithmic non-small cell carcinoma cells were inoculated into 96-well cell culture plate with 3,000 cells/well, and 100 μL culture medium were added to each well, it was put in the incubator at 37°C and 5% CO_2_ saturation humidity for 24 hours. The control group was only given the same volume of medium, and the combined group was cultured with the same number of non-small cell cancer cells. HA-Gd2O3-NPs of different concentrations (0, 15, 30, 45, 60 mg/L) were added, respectively, with 5 plates of each concentration, and then given different doses of irradiation (0, 3, 6, 9, 12 Gy). After treatment, they were placed at 37°C 5% CO2 saturation humidity incubator for 24 h, and 10 μL CCK-8 reagent was added to each well, continuing to incubate in the dark for 4 h, and measuring the optical density value (D value) of each well at the wavelength of 490 nm of the microplate reader. Six parallel wells were set for each concentration, and the experiment was repeated three times. The inhibition rate of cell proliferation was calculated according to the following equation.

(2) $$Cell\;proliferation\;inhibition\;rate=1-\frac{D\;value\;of\;union\;group}{D\;value\;of\;control\;group}\times 100\%$$

### 2.6 Efficacy evaluation index

The short-term efficacy was evaluated by response evaluation criteria in solid tumors (RECIST) [14], which was divided into four types: complete remission (CR), partial remission (PR), shakedown (SD), and proceeding (PD). CR means that all visible lesions disappeared and all lymph nodes were reduced to less than 10 mm and maintained for at least 4 weeks. PR means that the sum of the maximum diameters of all target tumor foci is reduced by more than 30% compared with the baseline level and maintained for at least 4 weeks. PD means that the sum of the maximum diameters of all target tumors increases by more than 20% compared with the minimum, and the absolute value of the increase of the longest diameter is at least 5 mm, or one or more new lesions appear. SD indicates between partial remission and proceeding. The short-term overall response rate (ORR) equation is as follows:

(3) $$ORR=\frac{CR+PR}{The\;total\;number\;of\;cases}\times 100\%$$

The adverse reactions were evaluated using the Common Terminology Criteria for Adverse Events (CTCAE4.0) of the National Cancer Institute and the classification standard of the Radiation Therapy Oncology Group (RTOG) [15]. The incidence and grade of adverse events including bone marrow suppression, liver function injury, diarrhea, rash, nausea, vomiting, acute radiation pneumonia, and acute central nervous system adverse reactions were statistically analyzed. The progression-free survival (PFS) and one-year survival rate were used to evaluate the long-term efficacy from the beginning of admission to the end of follow-up. The tumor markers in the two groups were statistically analyzed: cytokeratin 19 fragment (CYFRA21 – 1) and neuron-specific enolase (NSE).

RETRACTED

### 2.7 Follow-up

By means of outpatient review, wechat or telephone interview, the patients were followed up every 2 months within 1 year after the treatment, and then every 6 months. The follow-up was terminated in April 2021.

### 2.8 Statistical methods

The data of this study were analyzed by SPSS19.0 statistical software. All data were expressed by mean ± standard deviation ($\overset{ˉ}{x}$±s), and the counting data were expressed by frequency and percentage (%). The differences of general data, incidence of adverse reactions, and one-year survival rate before treatment were compared by chi-square test, and the differences of short-term efficacy were analyzed by rank sum test. The difference was statistically significant (*P <* 0.05).

## 3. Results

### 3.1 Study purpose and work content

The purpose of this study was to investigate the clinical efficacy and safety of EGFR-TKI targeted drugs combined with HA-Gd2O3-NPs in non-small cell lung cancer (NSCLC). 70 patients with stage IV EGFR mutant NSCLC were selected. They were randomly divided into combined group (35 cases) and control group (35 cases). HA-Gd2O3-NPs were prepared by hydrothermal polyol method and combined with epidermal growth factor receptor tyrosine kinase receptor inhibitor in the clinical treatment of NSCLC. The phase composition, morphology, and particle size distribution of HA-Gd2O3-NPs were observed. After EGFR-TKI resistance, patients in the control group only received chemotherapy. After EGFR-TKI resistance, patients in the combined group received three-dimensional conformal radiation EGFR-TKI targeted drug therapy. Statistical analysis included the incidence and grade of adverse events such as bone marrow suppression, liver function injury, diarrhea, rash, nausea, vomiting, acute radiation pneumonia and acute central nervous system adverse reactions. The long-term efficacy was evaluated by tumor progression-free survival and 1-year survival rate from the beginning of enrollment to the end of follow-up. Statistics of tumor markers in two groups: cytokeratin 19 fragment and transmembrane-specific enolase. By means of outpatient review, wechat or telephone interview, the patients were followed up every 2 months within 1 year after the treatment, and then every 6 months.

RETRACTED

### 3.2 Physical and chemical characteristics of hyaluronic acid-gadolinium trioxide-nanoparticles

HA-Gd2O3-NPs were successfully constructed by hydrothermal polyol method using hyaluronic acid, gadolinium chloride, and passivation molecules. The morphology of hyaluronic acid gadolinium trioxide nanoparticles was characterized by transmission electron microscope. It showed that they were spherical, uniform particle size, about 124 nm, and had good water solubility and dispersion; it can improve the bioavailability of targeted drugs. X-ray diffraction patterns show that hyaluronic acid gadolinium trioxide nanoparticles have two wide diffraction peaks at 5 ° and 30 °, respectively, indicating that the nanoparticles have poor crystal structure. The average entrapment efficiency of HA-Gd2O3-NPs was 90.31%. Figure 2 shows the physicochemical characteristics of hyaluronic acid gadolinium trioxide nanoparticles.

**Figure 2.** Physicochemical characteristics of hyaluronic acid gadolinium trioxide nanoparticles.A: electron microscopy B: particle size distribution C: X-ray diffraction pattern

### 3.3 Effect of hyaluronic acid-gadolinium trioxide-nanoparticles on cell proliferation inhibition rate

The experimental results of non-small cell lung cancer showed that the proliferation inhibition rates of 0, 15, 30, 45, and 60 mg/L hyaluronic acid gadolinium trioxide nanoparticles on NSCLC cells were 0%, 0.651%, 3.814%, 4.952%, and 4.126%, respectively. The inhibition rate of hyaluronic acid gadolinium trioxide nanoparticles on the proliferation of NSCLC cells increased gradually with the increase of mass concentration, and the inhibition rates of each concentration were less than 5%. There was no significant difference between the groups (*P >* 0.05). The above data show that hyaluronic acid gadolinium trioxide nanoparticles have no significant effect on the activity of NSCLC cells (Figure 3).

**Figure 3.** Effects of different concentrations of hyaluronic acid-gadolinium trioxide-nanoparticles on cell proliferation inhibition rate

### 3.4 Effect of hyaluronic acid-gadolinium trioxide-nanoparticles on lung tissue morphology

The results of hematoxylin–eosin staining showed that NSCLC cells were chrysanthemum-like and glandular in morphology. The cells were small and the size was relatively consistent. The cells were more diffusely distributed. Some were cord-like, necrotic, and neutrophilic. There was no obvious morphological change in the histology of the control group and the combined group, and no obvious inflammatory reaction was found, indicating that hyaluronic acid-gadolinium trioxide-nanoparticles had no obvious toxic and side effects on lung tissue (Figure 4).

RETRACTED

**Figure 4.** HE staining results. (a) normal lung tissue cells. (b) the study group organized cells after radiotherapy (c) tissue cells of control group after treatment

### 3.5 Radiosensitization effect of hyaluronic acid-gadolinium trioxide-nanoparticles

Under X-ray irradiation, with the increase of hyaluronic acid-gadolinium trioxide-nanoparticles concentration (0–60 mg/L) or radiation dose (0–9 Gy), the inhibition rate of non-small cell cancer cells was significantly increased. Especially, the survival rate of 45 mg/L non-small cell cancer cells under 6 Gy X-ray irradiation was the lowest of 66%, indicating that hyaluronic acid-gadolinium trioxide-nanoparticles had radiosensitization effect.

In order to verify the toxic effect of hyaluronic acid-gadolinium trioxide-nanoparticles on non-small cell cancer cells, 45 mg/L hyaluronic acid-gadolinium trioxide-nanoparticles were selected according to the results of cell viability CCK-8 under 6 Gy X-ray irradiation. The data showed that hyaluronic acid-gadolinium trioxide-nanoparticles had no toxic and side effects on non-small cell cancer cells. The cell survival rate of nonsmall cell cancer cells in the combined group was 37.2 ± 5.3%, and that of the control group was 98.4 ± 12.6% under 6 Gy X-ray irradiation, indicating that hyaluronic acid-gadolinium trioxide-nanoparticles had good radiosensitization function (Figure 5).

**Figure 5.** Effect of hyaluronic acid-gadolinium trioxide-nanoparticles on the activity of non-small cell cancer cells

A: effects of different concentrations of hyaluronic acid-gadolinium trioxide-nanoparticles on the activity of non-small cell cancer cells under different X-ray dosesB: effect of hyaluronic acid-gadolinium trioxide-nanoparticles on the activity of non-small cell cancer cells in two groups of patients* represents a statistical difference compared with the control group (*P <* 0.05)

### 3.6 Comparison of general data between the two groups of patients

There was no significant difference in the age, gender, pathological type, smoking history, PS score, and other general data of the two groups (*P >* 0.05). Figure 6a shows the comparison of the general data of the two groups.
**Figure 6a.** Comparison of general data between the two groups. (a) age comparison (b) gender comparison (c) comparison of pathological types (d) comparison of smoking history (e) PS score comparison

**Figure 6b.** continued

### 3.7 Comparison of short-term efficacy between the two groups of patients

The partial remission rate in the control group (17.14%) was significantly lower than that in the study group (42.86%). The shakedown rate of the control group (68.57%) was significantly higher than that of the study group (22.86%). The total effective rate of the control group (20%) was significantly lower than that of the study group (42.86%). There were significant differences in the above data (*P <* 0.05). There was no significant difference in other data (*P >* 0.05). Figure 7 shows the comparison of short-term curative effects between the two groups.

RETRACTED

**Figure 7.** Comparison of short-term efficacy between the two groups of patients

Note: * represents a statistical difference compared with the control group (*P <* 0.05)

### 3.8 Comparison of one-year survival rate between the two groups of patients

The one-year survival rate of the combined group (94%) was significantly higher than that of the control group (75%) (*P <* 0.05) (Figure 8).

**Figure 8.** Comparison of one-year survival rates between the two groups of patients

* represents a statistical difference compared with the control group (*P <* 0.05)

### 3.9 Comparison of progression-free survival between the two groups of patients

The median progression-free survival was 8 months in the control group and 12 months in the combined group, with statistical difference (*P <* 0.05). Figure 9 is comparison of progression-free survival between the two groups.

**Figure 9.** Comparison of progression-free survival between the two groups of patients

### 3.10 Comparison of tumor marker levels between the two groups

The CYFRA21 – 1 level in the control group (3.8 ± 0.4 μg/L) was significantly higher than that in the combined group (2.3 ± 0.2 μg/L), with statistical difference (*P <* 0.05). The NSE level of the control group (21.5 ± 1.3 μg/L) was significantly higher than that of the combined group (13.4 ± 1.2 μg/L), with statistical difference (*P <* 0.05) (Figure 10).

**Figure 10.** Comparison of tumor marker levels between the two groups

*indicates that there is a statistical difference compared with the control group (*P <* 0.05)

### 3.11 Comparison of adverse events between the two groups

There were 11 cases (31.43%) of bone marrow suppression in the combined group and 10 cases (28.57%) in the control group. There were 5 cases (14.29%) of liver function injury in the combined group and 6 cases (17.14%) in the control group. There were 12 cases (34.29%) of rash in the combined group and 9 cases (25.71%) in the control group. There was 1 case (2.86%) of diarrhea in the combined group and 2 cases (5.71%) in the control group. There were 15 cases (42.86%) of nausea and vomiting in the combined group and 6 cases (17.14%) in the control group, with statistical difference (*P <* 0.05) (Figure 11).

RETRACTED

**Figure 11.** Comparison of adverse events between the two groups

* indicates that there is a statistical difference compared with the control group (*P <* 0.05)

## 4. Discussion

At present, prolonging the survival time of patients with NSCLC is a global problem. The treatment of NSCLC patients with traditional platinum-based dual-drug chemotherapy has reached the plateau stage. Increasing the dose of chemotherapy drugs cannot improve the clinical efficacy, but also increase the incidence of adverse reactions, and the quality of life of patients is reduced. High-dose and long-term radiotherapy will increase the probability of radiation damage [16,17]. In contrast, targeted drug therapy can accurately act on the carcinogenic sites of cancer cells, killing tumor cells specifically, not only reduces the damage to normal tissues around the lesion, but also improves the accuracy of killing tumor cells [18]. Heavy metal nanoparticles (Au, Pt, Gd, etc.) have X-ray photon capture cross-section effect, and their dose sensitization can significantly provide radiation damage to sensitive target cells. When heavy metal nanoparticles and photon energy act in tumor cells, the release of electrons will damage tumor cells and have good therapeutic effect.

The hyaluronic acid-gadolinium trioxide-nanoparticles prepared in this study are an effective radiosensitizer. The defects of vascular system and lymphatic drainage system in patients with NSCLC will lead to the gradual increase of endothelial gap and the increase of selective permeability of nanoparticles, which will produce high permeability effect. Due to the passive targeting effect of EGFR, nanomaterials with suitable sizes can aggregate in tumor sites, thus playing a role in the treatment of tumors. The particle size of hyaluronic acid-gadolinium trioxide-nanoparticles prepared in this experiment is about 124 nm and the size is uniform, so it can produce a strong high permeability effect and accumulate in the tumor site. Gd_2_O_3_ modified by hyaluronic acid has good water solubility and biocompatibility. It is necessary to detect the effect of hyaluronic acid-gadolinium trioxide-nanoparticles on cell activity and lung. Wang et al. (2019) [19] pointed out that nano materials between 100 and 200 nm are more likely to be ingested by solid tumors. In this study, it was found that 60 mg/L hyaluronic acid-gadolinium trioxide-nanoparticles had no significant effect on the cell activity of NSCLC cells, which was similar to the study of Song et al. (2020) [20]. In addition, hyaluronic acid-gadolinium trioxide-nanoparticles can significantly inhibit the proliferation of NSCLC cells under X-ray irradiation, which has a certain radiosensitization effect. Therefore, radiotherapy combined with hyaluronic acid-gadolinium trioxide-nanoparticles has a certain application prospect in the treatment of NSCLC.

RETRACTED

EGFR-TKI targeted drug therapy cannot coexist with surgical treatment. When EGFR gene mutation occurs in patients with advanced NSCLC, EGFR-TKI targeted drug therapy is the first-line standard treatment. EGFR belongs to the plasma membrane receptor tyrosine kinase family, which can regulate the proliferation and apoptosis of tumor cells. If EGFR is activated in tumor cells, it will lead to accelerated tumor proliferation and easy invasion and metastasis. About 85% of patients with NSCLC had high EGFR expression in lung adenocarcinoma and lung squamous cell carcinoma. Nowadays, the biggest problem facing oncology is that patients with NSCLC will have resistance to EGFR-TKI targeted drugs after EGFR mutation. In order to improve the clinical efficacy of EGFR-TKI targeted drugs, studies have proposed EGFR-TKI targeted combination therapy [21,22]. HA-Gd2O3-NPs is nontoxic in normal cells, but has obvious uptake behavior in drug-resistant cells, which improves the concentration of drugs in cells to a certain extent, enhances the cytotoxicity of drugs and improves the therapeutic effect. EGFR-TKI targeted combination therapy group is better than the control group, which may be related to the synergy between EGFR-TKI targeted drugs and combination therapy. The results showed that the total effective rate, 1-year survival rate, and progression-free survival in the EGFR-TKI combined group were better than those in the single control group. The levels of tumor markers CYFRA21-1 and NSE in the control group were significantly higher than those in the combined group (*P <* 0.05). The incidence of nausea and vomiting in the combined group was higher than that in the control group (*P <* 0.05). There was no significant difference in the incidence of other adverse reactions such as diarrhea, rash, liver function injury, and bone marrow suppression between the combined group and the control group (*P >* 0.05).

## 5. Conclusion

In this study, HA-Gd2O3-NPs were prepared and combined with epidermal growth factor receptor tyrosine kinase receptor inhibitor in the clinical treatment of NSCLC. EGFR-TKI targeted drugs combined with HA-Gd2O3-NPs can significantly improve the clinical efficacy and survival of patients with stage IV EGFR mutant NSCLC. The deficiency of this study is the small sample size. In the future, we need to expand the sample size and increase multi-center research to further verify the experimental conclusions, so as to provide more clinical treatment schemes for clinical treatment of NSCLC.
